# Risk Factors and Distribution Characteristics of Intracranial and Intracranial Artery Stenosis in Young Sufferers with Ischemic Stroke

**DOI:** 10.1155/2022/9684158

**Published:** 2022-06-24

**Authors:** Yongchao Wang, Yan Wei

**Affiliations:** Department of Neurology, Hengshui People's Hospital, Hengshui 053000, China

## Abstract

In order to explore the risk factors of intracranial and intracranial arterial stenosis, the distribution of young ischemic stroke sufferers with intracranial and intracranial arterial stenosis and the related are analyzed. In this study, a total of 213 young sufferers with ischemic stroke (IS) admitted to our hospital from February 2019 to September 2021 are selected. According to the CT diagnosis of intracranial artery stenosis (AS), 213 patients are divided into two groups, with 86 in the AS Group and 127 in the non-AS Group. To analyze the distribution of intracranial and intracranial AS in young patients with ischemic stroke, 86 patients with AS are examined by carotid B-mode ultrasound. Furthermore, a univariate analysis is performed on the relevant indicators of the sufferers in the cancer (CA) set and the two sets without CA, and then, the indicators with statistically extensive disparity were selected for multivariate logistic regression analysis of the risk factors for CA symptoms. The results show 50% of the sufferers with moderate or severe ischemic CA in young adults and 63.95% of the sufferers with intracranial artery stenosis. It is clearly evident that the main risk factors affecting the occurrence of intracranial and intracranial arteries in young IS are hypertension and long-term smoking, long-term drinking, and hyperlipidemia.

## 1. Introduction

Ischemic stroke (IS) is a cerebrovascular disease caused by cerebral ischemia, hypoxia, necrosis, softening, and infarct formation due to blood supply disorder in the brain [1]. As one of the cerebrovascular diseases with high clinical incidence rate, the incidence rate of adolescents is gradually rising [2]. Research shows that in patients with ischemic stroke, the proportion of patients with cerebral artery stenosis is about 30%–50%, and the proportion of AS in young patients with ischemic stroke is 1/3 [3, 4]. It should be noted that the morbidity and mortality of stroke sufferers with symptoms of intracranial and extracranial arteriostenosis seriously threaten the health and safety of young people [5]. At present, the examination methods used in young IS sufferers with AS have different advantages and disadvantages. Arterial stenosis usually occurs in carotid artery, intracranial artery, and coronary artery. Some patients may also have lower extremity arterial stenosis. The main cause of arterial stenosis is atherosclerosis, as well as arteritis and aortic dissection. Under the inducement of hyperlipidemia, hypertension, and hyperglycemia, arterial elasticity decreases with age and arteriosclerosis gradually forms. If the atherosclerotic plaque is not well controlled, plaque proliferation may cause lumen stenosis. If the stenosis is serious and the blood flow speed is slow, thrombosis may be formed in the blood vessels. However, digital subtraction angiography (DSA) of the whole brain is unified as the “golden gold” for diagnosing the occurrence of AS in young IS sufferers [6, 7]. The reason is that DSA can clearly show the distribution site and stenosis degree of AS and provide diagnostic criteria for subsequent therapy. Some studies have shown that [8] the probability of AS symptoms in young ischemic stroke sufferers accounts for an extensive proportion and there is no unified conclusion on the distribution characteristics and risk factors of young ischemic stroke sufferers with intracranial and intracranial arterial stenosis. Analysis of the risk factors and distribution characteristics of AS symptoms in young ischemic stroke sufferers is of great significance to improve the prognosis of IS sufferers and reduce the mortality of sufferers [9, 10]. However, the distribution characteristics and pathogenic factors of cerebral artery stenosis in young IS sufferers are not clear [11, 12].

Therefore, this paper takes young sufferers with IS as the research subject and analyzes the risk factors and distribution characteristics of intracranial and intracranial artery stenosis in young sufferers with ischemic stroke.

The remainder of this paper is organized as follows.  Section 2 discusses the related work, followed by the general information and methods in Section 3. The results and analysis is discussed in Section 4.  Section 5 concludes the paper with a summary.

## 2. Related Work

Cerebrovascular accident (CVA) is one of the common diseases of acute cerebrovascular diseases, which is clinically known as “stroke” [13]. The main cause of stroke is the sudden rupture of blood vessels in the patient's brain. It can cause blockage and prevent blood flow to the brain, which causes tissue damage to the brain [14]. The most common symptom of stroke is arterial embolism after the small embolus on the inner wall of cerebral blood supply vessel falls off, that is, ischemic stroke. With age, the symptoms of AS will be a chronic noninflammatory vascular disease. It is characterized by arterial wall thickening and severe lumen stenosis, resulting in lumen obstruction [15]. Relevant research on intracranial artery stenosis or occlusion [16] showed that the rate of intracranial artery stenosis in IS sufferers was as high as 47%. Cerebral artery stenosis is one of the most common causes of IS. Many studies have shown that ischemic stroke caused by intracranial artery stenosis has a higher risk of recurrent stroke than other types of ischemic stroke, especially for sufferers with multiple intracranial stenosis [17, 18].

The number of people with a family history of cerebrovascular disease is also higher than the set without AS symptoms. The reason is that the lipids of sufferers with hyperlipidemia are deposited in the blood vessel wall. It results in the formation of atherosclerotic plaques and vascular stenosis and promotes thrombosis [19–21]. Long-term smoking will disturb the lipid metabolism in the body, increase blood viscosity, and eventually cause platelets to aggregate, causing symptoms of intracranial and intracranial arterial stenosis [22, 23]. Therefore, drinking and smoking, living habits for more than 3 years, sufferers with hypertension, hyperlipidemia, and other cerebrovascular diseases are the pathogenic factors that induce AS symptoms in sufferers. Clinical studies have shown that cerebral arterial stenosis is dominated by anterior circulation lesions, and the incidence of intracranial arterial stenosis is higher than that of extracranial arteries. The results of our study showed that 43 cases of stenosis were distributed in the anterior circulation of intracranial artery stenosis, accounting for 50%, and 12 cases were distributed in the circulation after intracranial artery stenosis, accounting for 13.95%, and the incidence of intracranial artery stenosis was the highest, accounting for 63.95%. Also, it can be observed that the intracranial artery stenosis in the sufferers with juvenile ischemic stroke was distributed in 11 sufferers with PCA (accounting for 20%) and 12 sufferers with VA (accounting for 22%). The main distribution sites of internal artery stenosis were in MCA and VA. 12 sufferers with extracranial artery stenosis were located in E-ICA (accounting for 39%) and 10 sufferers were in E-VA (accounting for 33%). Extracranial artery stenosis was mainly distributed in E-ICA. For ICA and E-VA, the analysis may be due to different factors such as personal living habits and the location of stenosis is also different. Some studies have pointed out that the elderly with smoking history generally have hypertension, diabetes, coronary heart disease, and hyperlipidemia. For young IS sufferers, the developing intracranial and intracranial arterial stenosis are high-risk factors [18]. The multivariate analysis of intracranial and intracranial artery stenosis in young sufferers with ischemic stroke by a logistic multiple regression equation shows that the survey content of the two sets of young IS sufferers showed that there were more than 3 years of smoking and more than 3 years of drinking. The number of habitual sufferers with intracranial and intracranial arterial stenosis was notoriously higher than the number without intracranial and intracranial arterial stenosis. Comparing the clinical data of the two sets of sufferers found that young ischemic sufferers with AS symptoms suffered from hypertension, hyperlipidemia, and concomitant complications.

## 3. General Information and Methods

### 3.1. General Information

213 young IS patients admitted to our hospital from February 2019 to September 2021 were taken as the research subjects, and 213 patients were divided into two groups according to whether AS occurred. There were 86 cases in the AS Group, including 69 males (80.23%) and 17 females (17.44). Their ages ranged from 19 to 41 years, and the average age was (28.99 ± 4.49) years. The course of the disease was 3 to 7 weeks. In addition, there were 127 patients in the non-AS Group, including 77 males (60.63%) and 50 females (39.37%). Their ages ranged from 21 to 15 years old, the average age was (30.44 ± 3.09), and the course of disease was 2 to 8 weeks. There was no significant difference between the two groups in general data such as age and male female ratio (*P* > 0.05).

Inclusion criteria include the following conditions: (1) the age of the sufferers is 18–50 years old; (2) meet the clinical diagnostic criteria; (3) have no other chronic diseases; (4) have good understanding and communication skills; and (5) have no history of mental illness.

Exclusion criteria include the following conditions: (1) cardiogenic embolism; (2) severe failure of organs such as liver and kidney; (3) sufferers with malignant tumors; (4) sufferers with other vascular diseases; and (5) venous system infarction.

All the sufferers participating in the study had a detailed understanding of the content and purpose of the study, obtained the sufferer's consent, and signed an informed consent form.

### 3.2. Methods

Brain MRI, magnetic resonance angiography, and color Doppler ultrasound of bilateral carotid and vertebral arteries were performed for the two sets of sufferers. According to the data of head imaging, the sufferers were divided into a AS set and a non-AS set. All 86 sufferers underwent femoral artery puncture DSA examination to observe the distribution of AS in the sufferers. For example, the self-made questionnaire was used to investigate the daily life habits and clinical data of the two sets of sufferers, and the sufferers were informed that they should keep an empty stomach in the early morning on the first day of admission, in order to test blood sugar and blood lipids. The results of brain magnetic resonance imaging, magnetic resonance angiography, bilateral carotid artery, and vertebral artery color Doppler ultrasound and DSA examination results were collected after admission. The comparison of the diameter of the stenosis at this segment with the adjacent normal diameter is less than 50% or the whole branch of the artery is not visualized, which can be considered as stenosis or occlusion of the blood vessel. The degree of stenosis can be calculated by the formula: Degree of stenosis = (1 − Remaining lumen)/Total lumen *x* 100%. According to the North American Symptomatic Carotid Endarterectomy Trial research method, the degree of vascular stenosis was divided into several categories: mild stenosis (<50%), moderate stenosis (50%–69%), severe stenosis (70%–99%), and occlusion (100%).

### 3.3. Observation Indicators and Evaluation Criteria

1. Judgment criteria for intracranial and extracranial arterial stenosis: Cranial magnetic resonance angiography shows that the blood vessels of this segment are continuously displayed throughout the whole process, with clear and sharp edges, basically uniform signals, and no dislocation phenomenon, and it can be considered that the blood vessels have no stenosis.
2. Ultrasound was used as a reference for the location and degree of vascular stenosis, and DSA was used as the gold standard when the results were inconsistent.
3. The clinical data of the two sets of sufferers were recorded in detail. In the self-made questionnaire of our hospital, the long-term smoking time was defined as ≥10 cigarettes/d for more than 3 consecutive years; long-term drinking was drinking ≥60 g/d for more than 3 consecutive years; staying up late is defined as sleeping after 1 a.m. every day for more than a year.
4. The clinical data of the two sets of sufferers were analyzed by univariate analysis, and the relevant factors with statistically extensive disparity at *P* < 0.05 were selected.
5. logistic multiple regression equation was used to analyze the risk factors of intracranial and intracranial arterial stenosis in sufferers with multiple factors.

### 3.4. Statistical Processing

SPSS 24.0 software was used for statistical processing. Measurement data were expressed as mean ± standard deviation ($\bar{x}$ ± *s*), and two independent samples' *t*-test was used for comparison between sets. Counting data were subjected to *χ*^2^ test, expressed in %, and *P* < 0.05 was considered statistically extensive. Whether the sufferers had long-term smoking, long-term drinking, long-term staying up late, diabetes, hypertension, hyperlipidemia, and family history of cerebrovascular disease were counted. The logistic multiple regression equation was used to analyze the risk factors of IS among AS youths. *P* < 0.05 was considered statistically extensive.

## 4. Results and Analysis

### 4.1. Degree of Lumen Stenosis in Sufferers with AS Symptoms

Among the 86 sufferers with AS, 32 had mild stenosis, accounting for 37.21%, 43 had moderate or severe stenosis, accounting for 50%, and 11 had intracranial artery occlusion, accounting for 12.799%, as shown in Table 1 and Figure 1.

### 4.2. Stenosis Distribution of Sufferers with AS

Among the 86 sufferers with AS, 43 cases of stenosis were distributed in the anterior circulation of intracranial artery stenosis, accounting for 50%, 14 cases were distributed in the anterior circulation of extracranial artery stenosis, accounting for 16.28%, and 12 cases were distributed in the intracranial artery. The post-stenosis circulation accounted for 13.95% and the 17 cases distributed in the extracranial artery post-stenosis accounted for 19.77%, as shown in Table 2 and Figure 2.

### 4.3. Distribution of Intracranial Stenosis in Sufferers with AS Symptoms

The results of intracranial artery stenosis distribution showed that 4 sufferers had intracranial artery stenosis at I-ICA (accounting for 7%), 6 sufferers were at ACA (accounting for 11%), and 18 sufferers were at MCA (accounting for 33%). There are 4 sufferers with BA (accounting for 7%), 11 sufferers with PCA (accounting for 20%), and 12 sufferers with VA (accounting for 22%). Besides, the incidence of intracranial artery stenosis is higher in MCA and VA as shown in Table 3 and Figure 3.

### 4.4. Distribution of Extracranial Stenosis in Sufferers with AS Symptoms

The results of intracranial artery stenosis distribution showed that 5 sufferers had extracranial artery stenosis at CCA (accounting for 16%), 4 sufferers were at SCA (accounting for 13%), and 12 sufferers were at E-ICA (accounting for 39%). There were 10 sufferers with E-VA, accounting for 33%; the distribution of extracranial artery stenosis was higher in E-ICA and E-VA as shown in Table 4 and Figure 4.

### 4.5. Univariate Analysis of the Living Habits of the Two Sets of Sufferers

After univariate analysis, the number of long-term smokers and long-term drinkers in the AS symptom set was notoriously higher than that in the non-AS set (*P* < 0.05), and the disparity was statistically extensive as shown in Table 5.

### 4.6. Univariate Analysis of the Clinical Data of the Two Sets of Sufferers

The results of univariate analysis showed that the number of hypertension, hyperlipidemia, and cerebrovascular family history in the AS symptom set was higher than that in the non-AS set (*P* < 0.05) and the disparity was statistically extensive as shown in Table 6.

### 4.7. Logistic Analysis of Risk Factors in Young Ischemic Stroke Sufferers with AS Symptoms

The multivariate analysis assignment scale is shown in Table 7. The incidence of ischemic stroke in young people with AS symptoms is used as the research dependent variable, and long-term smoking, long-term drinking, hypertension and hyperlipidemia, and history of cerebrovascular disease are used as independent variables. The model was selected based on the actual clinical situation. The results of logistic regression model analysis showed that long-term smoking, long-term drinking, hypertension, hyperlipidemia, and history of cerebrovascular disease were the risk factors for ischemic stroke in young people with AS symptoms (*P* < 0.05) as shown in Table 8.

## 5. Conclusions

In this study, risk factors and distribution characteristics of intracranial and intracranial artery stenosis in young sufferers with ischemic stroke were investigated. The results of our study demonstrate that the proportion of young stroke sufferers with intracranial and intracranial artery stenosis is higher in sufferers with intracranial artery stenosis than in extracranial arteries, especially in MCA and VA. The number of sufferers with ICA and E-VA is relatively extensive, and the risk factors for the occurrence of intracranial and intracranial artery stenosis in young stroke sufferers are mainly those with hypertension, hyperlipidemia, longer smoking age, and long-term drinking.

This study has made some achievements, but there are still some limitations. Due to the small sample size and only the young ischemic stroke patients in this region and our hospital as the research subject, different risk factors in different regions were not fully considered. In future research, we will expand the sample size and comprehensively analyze the harm of various risk factors to patients.

## Figures and Tables

**Figure 1:** Characteristic map of the degree of lumen stenosis in sufferers with AS symptoms.

**Figure 2:** Distribution of AS in sufferers.

**Figure 3:** Distribution of intracranial artery stenosis in sufferers.

**Figure 4:** Distribution of extracranial artery stenosis in sufferers.

**Table 1:** Characteristics of the degree of lumen stenosis in sufferers with AS symptoms.

Stenosis	Number of cases (*n* = 86)	Percentage (%)
Mild stenosis	32	37.21
Moderate to severe stenosis	43	50.00
Occlusion	11	12.79

**Table 2:** Distribution of AS in sufferers.

Narrow distribution	Number of cases (*n* = 86)	Percentage (%)
Intracranial artery stenosis precirculation	43	50.00
Circulation after intracranial artery stenosis	14	16.28
Extracranial artery stenosis precirculation	12	13.95
Circulation after extracranial artery stenosis	17	19.77

**Table 3:** Distribution of intracranial artery stenosis in sufferers.

Distribution of intracranial artery stenosis	Number of cases (*n* = 55)	Percentage (%)
I-ICA	4	0.05
ACA	6	0.11
MCA	18	0.33
BA	4	0.07
PCA	11	0.20
VA	12	0.22

**Table 4:** Distribution of extracranial artery stenosis in sufferers.

Distribution of extracranial artery stenosis	Number of cases (*n* = 33)	Percentage (%)
CCA	5	0.16
SCA	4	0.13
E-ICA	12	0.39
E-VA	10	0.33

**Table 5:** Comparison of living habits of the two sets of sufferers.

Set	Smoking for more than 3 years (%)	Drinking alcohol for more than 3 years (%)	Stay up late for more than a year (%)
AS (*n* = 86)	44 (51.16)	32 (37.21)	10 (11.62)
Non-AS set (*n* = 127)	30 (23.62)	21 (16.54)	76 (59.82)
*x* ^2^	4.372	2.031	1.147
*P*	0.004	0.044	0.539

**Table 6:** Comparison of clinical data of two sets of sufferers.

Set	Hypertension (%)	Hyperlipidemia (%)	Cerebrovascular family history (%)	Diabetes (%)
AS (*n* = 86)	34 (39.53)	30 (34.88)	9 (10.47)	11 (12.79)
Non-AS set (*n* = 127)	20 (15.75)	12 (9.00)	5 (4.00)	90 (69.77)
*x* ^2^	4.372	2.031	1.147	2.455
*P*	0.002	0.024	0.049	0.054

**Table 7:** Multivariate analysis assignment scale.

Factor	Assign
Dependent variable	Happened = 1; did not happen = 2
Induced AS symptoms in young ischemic stroke	
Independent variable	

Long-term smoking	yes = 1; no = 2
Long-term drinking	yes = 1; no = 2
Hypertension	Yes = 1; No = 2
Hyperlipidemia	Yes = 1; No = 2
History of cerebrovascular disease	Yes = 1; No = 2

**Table 8:** Logistic analysis of risk factors for inducing AS symptoms.

Factor	Β value	Wald value	*S. E*. value	*P* value	OR value
Long term smoking	0.197	10.263	0.146	0.016	4.005 (1.311∼4.716)
Long term drinking	0.203	11.504	0.527	0.021	2.963 (0.198∼3.340)
Suffering from hypertension	0.141	10.513	0.651	0.031	2.441 (1.237∼3.298)
Suffering from hyperlipidemia	1.246	9.247	1.413	0.017	0.500 (0.579∼1.296)
History of cerebral blood disease	1.271	10.418	1.433	0.033	2.113 (1.154∼3.048)

## Data Availability

The experimental data used to support the findings of this study are available from the corresponding author upon request.
